# Exploring the Active Ingredients and Mechanism of Action of Huanglian Huazhuo Capsule for the Treatment of Obese Type-2 Diabetes Mellitus Based on Using Network Pharmacology and Molecular Docking

**DOI:** 10.1155/2022/2780647

**Published:** 2022-10-03

**Authors:** Na Wang, Wen-bo An, Nan Zhou, Jing-chun Fan, Xin Feng, Wei-jie Yang

**Affiliations:** ^1^Gansu University of Chinese Medicine, Lanzhou, China; ^2^Affiliated Hospital of Gansu University of Chinese Medicine, Lanzhou, China; ^3^School of Public Health, Gansu University of Chinese Medicine, Lanzhou, China; ^4^Department of Endocrinology, Affiliated Hospital of Gansu University of Chinese Medicine, Lanzhou, China

## Abstract

**Background:**

Obese type 2 diabetes mellitus (obese T2DM) is one of the prime diseases that endangers human health. Clinical studies have confirmed the ability of the Huanglian Huazhuo capsule to treat obese T2DM; however, its mechanism of action is still unclear. In this study, effects and mechanisms of the Huanglian Huazhuo capsule in obese T2DM were systematically investigated using network pharmacology and molecular docking techniques.

**Methods:**

The active ingredients and targets of the Huanglian Huazhuo capsule were extracted from Traditional Chinese Medicine Systems Pharmacology Database and Analysis Platform (TCMSP). Obese T2DM diabetes-related targets were retrieved from a geographic dataset combined with a gene card database. A protein-protein interaction (PPI) network was constructed to screen core targets. The Gene Ontology (GO) and Kyoto Encyclopedia of Genes and Genomes (KEGG) pathway enrichment analyses were conducted using Database for Annotation Visualization and Integrated Discovery (DAVID). Interactions between potential targets and active compounds were assessed using molecular docking. Molecular docking was performed on the best core protein complexes obtained using molecular docking.

**Results:**

A total of 89 and 108 active ingredients and targets, respectively, were identified. Seven core targets were obtained using a topological analysis of the PPI network. The GO and KEGG pathway enrichment analyses showed that the effects of the Huanglian Huazhuo capsules were mediated by inflammation, lipid response, oxidative stress-related genes, and HIF-1 and IL-17 signaling pathways. Good binding ability was observed between the active compounds and screened targets using molecular docking.

**Conclusions:**

The active ingredients, potential targets, and pathways of the Huanglian Huazhuo capsule for the treatment of obese T2DM were successfully predicted, providing a new strategy for further investigation of its molecular mechanisms. In addition, the potential active ingredients provide a reliable source for drug screening in obese T2DM.

## 1. Introduction

Diabetes mellitus (DM) is a metabolic endocrine disease characterized by glucose and fat metabolism disorders and increased plasma glucose levels, and in the symptomatic stage, it is characterized by excessive drinking, polyphagia, polyuria, weakness, wasting, or sweet-tasting urine [1]. Relevant studies in recent years showed that the number of cases of obese type 2 diabetes mellitus (obese T2DM) with insulin resistance is gradually increasing. Obesity in such patients is primarily due to unreasonable diet structure and lack of exercise as well as the cause of insulin resistance [2], which are closely related. In addition, weight gain is an independent risk factor, particularly in central obesity, which predisposes to insulin resistance, leading to a high workload of pancreatic B cells and impaired islet function, resulting in lipolysis insulin inhibition [3].

In Chinese medicine, DM is not named but classifies as a “thirst disorder.” According to Traditional Chinese Medicine (TCM), the etiology of obese T2DM is complex, with congenital deficiency of endowment, emotional disorders, poor diet, and lack of exercise contributing to the disease. However, the congenital deficiency of endowment shows the most impact than others [4]. In the Huanglian Huazhuo capsule, Huanglian can clear away heat and dampness, stop diarrhea, and detoxify; Huangbai can clear away heat and dampness, purge fire, and detoxify; Danshen can activate blood circulation, remove blood stasis, and relieve pain; and Shanzha and Zhiqiao aurantii Immaturus can regulate qi, and relieve stagnation and swelling. Therefore, the Huanglian Huazhuo capsule has the functions of promoting qi and resolving phlegm, invigorating the spleen and eliminating accumulation, and removing dampness and blood stasis [5]. However, systematic studies on the mechanisms underlying the beneficial effects of the Huanglian Huazhuo capsule in T2DM are scarce, including the analyses of potential targets, biological processes, and metabolic pathways.

In Chinese medicine, traditional pharmacological approaches are limited to mechanistic studies [6]. In 2013, Shao Li proposed a new concept called “network pharmacology,” which provides a new strategy to determine the mechanism of action of herbal formulations [7]. Cyberpharmacology of TCM includes virtual computing, high-throughput data analysis, and web-based database search, involving bioinformatics network construction and network topology analysis [8]. This approach emphasizes multicomponent, multichannel, and multiobjective synergies and is well-suited for TCM analysis [8, 9]. Due to recent bioinformatics convergence, computational prediction-based network pharmacology is powerful to systematically reveal the biological mechanisms of complex diseases and drug effects at the molecular level [10, 11]. The potential mechanisms of TCM for the treatment of various diseases are increasingly studied using network pharmacology [12, 13]. Hence, major bioactive compounds, potential targets, and signaling pathways of the Huang Lian Huazhuo capsules were predicted using network pharmacology and molecular docking techniques in obese T2DM. The results provide the basis for investigating the mechanism of action of the Huanglian Huazhuo capsules in obese T2DM.

## 2. Materials and Methods

### 2.1. Data Collection

#### 2.1.1. Active Ingredients and Corresponding Targets of the Huanglian Huazhuo Capsule

The active components in the Huanglian Huazhuo capsule were retrieved using Traditional Chinese Medicine Systems Pharmacology Database and Analysis Platform (TCMSP, https://old.tcmsp-e.com/tcmsp.php). “Huanglian, Huangbai, Danshen, Shanzha, and Zhiqiao” were the keywords of the compound. Furthermore, the full name of the target gene was converted into an abbreviation. TCMSP is a systematic pharmacology platform for Chinese herbal medicine, providing interactive data associated with the relationship among drugs, targets, and diseases [14]. In addition, the platform provides data on chemical, target, and drug-target networks and pharmacokinetic effects, including drug similarity (DL), oral bioavailability (OB), intestinal epithelial permeability, water solubility, and blood-brain barrier permeability, of natural compounds. A comprehensive Traditional Chinese Medicine Integrated Database (TCMID, http://www.megabionet.org/tcmid/) provides data for TCM [15]. The OB and DL were ≥30% and ≥0.18, respectively [16], and the active compounds were further analyzed [17]. OB describes the delivery capacity of oral drugs to the systemic circulation [18], and DL is based on the similarities of several known drugs in functional groups and physical properties [19].

#### 2.1.2. Anti-Obese T2DM Targets of the Huanglian Huazhuo Capsule

The mRNA expression profile of an obese T2DM sample (GSE166467) was searched in the gene expression synthesis dataset (GEO: https://www.ncbi.nlm.nih.gov/GEO) [20]. The threshold for identifying differentially expressed genes (DEGs) using SVA and Limma packages in RStudio 4.2.1 (https://www.rstudio.com/products/rstudio/) was |log FC| > 1, *P* < 0.05 [21]. The DEGs were visualized to generate volcanic and thermal maps. Data on disease targets associated with obese T2DM are available in the GeneCards database (http://www.genecards.org/) [22] using the keyword “Obese T2DM” to screen disease genes and eliminate duplicate targets. The target intersection corresponding to the active ingredient and disease target was selected using Venny 2.1.0 (https://bioinfogp.cnb.csic.es/tools/venny/index.html), and the intersecting target was the action target of the Huanglian Huazhuo capsule in intervening obesity and diabetes.

#### 2.1.3. Constructing a “Drug-Component-Target-Disease” Network

The drugs, active ingredients, and intersection targets of drugs and diseases were input in the Cytoscape 3.8.0 software (https://cytoscape.org/). The network diagram of “drugs-component-targets-diseases” was constructed, which was analyzed using the cytoNCA plug-in.

#### 2.1.4. Construction and Analysis of Protein-Protein Interaction Network

The data of drug-disease intersection genes were imported to the STRING website (https://cn.string-db.org/). The species was restricted to “*Homo sapiens*,” and data with confidence levels higher than 0.90 were selected. The obtained data were imported into the Cytoscape 3.8.0 software for analysis, and graphs were generated by identifying the core genes of the network.

#### 2.1.5. GO and KEGG Enrichment Analyses

Drug-disease intersection targets were subjected to GO and KEGG analyses using the RStudio 4.2.1 package and bioconductor package (https://mirrors.tuna.tsinghua.edu.cn/bioconductor), respectively. Enrichment analysis statistical filter values were set (*P*=0.05, *Q* = 0.05), and the screening results were visualized.

#### 2.1.6. Construction of Compound-Target-Pathway Networks

Compound-target-pathways were constructed and analyzed using Cytoscape 3.8.0 to visualize and elucidate the complex associations among compounds, pathways, and targets.

#### 2.1.7. Prediction of the Binding Ability of the Huanglian Huazhuo Capsule Core Components to the Target Using Molecular Docking Technique

The 3D structure of the target protein was downloaded from the Research Collaboratory for Structural Bioinformatics, Protein Data Bank (RSCB PDB) database (http://www.rcsb.org), and the water and protein impurities were removed using PyMOL (https://pymol.org/) software. The 2D structure of the active ingredient was downloaded from the PubChem database (https://pubchem.ncbi.nlm.nih.gov/) and imported into Chem3D software (https://www.chemdraw.com.cn/) to convert it into a 3D structure. The target proteins and small molecules were hydrogenated using AutoDockTools 1.5.6 software (https://autodock.scripps.edu/). The Grid Box was set up with the original ligand as the center, and the data were derived, followed by AutoDock Vina application for molecular docking. The target proteins and small molecules were visualized using the PyMoL software.

## 3. Results

### 3.1. Active Ingredients and Corresponding Targets of the Huanglian Huazhuo Capsule

From the TCMSP database, 57 active ingredients of “Danshen,” 22 of “Huangbai,” 10 of “Huanglian,” 6 of “Shanzha,” and 5 of “Zhiqiao” were found in the Huanglian Huazhuo capsule after screening. A total of 88 active ingredients were selected after combining and de-weighting all the data (Table 1).

### 3.2. Differentially Expressed Genes in Obese T2DM

A total of 28 DEGs were identified from this series of analysis (GSE166467). Of these, 19 were upregulated and 9 were downregulated in the obese T2DM (Figure 1(a)). The heat map of the expression patterns of the 28 DEGs is shown in Figure 1(b).

### 3.3. Anti-Obese T2DM Action Targets of the Huanglian Huazhuo Capsule

A total of 222 active ingredient targets of the Huanglian Huazhuo capsule were identified using the TCMSP database, and 1056 genes associated with obese T2DM and 108 targets of the drug-disease intersection were obtained using the GeneCards database (Figure 2).

### 3.4. Construction of “Drug-Component-Target-Disease” Network

The “Drug-Component-Target-Disease” network of the Huanglian Huazhuo capsule was mapped using the Cytoscape 3.8.0 software for obesity and DM treatment (Figure 3(a)). The diagram consisted of 298 nodes and 1652 edges, with 88 active ingredients and 108 potential targets. The active components of the Huanglian Huazhuo capsule before the moderate value were quercetin, beta-sitosterol, stigmasterol, kaempferol, luteolin, tanshinone IIA, and naringenin. Furthermore, these seven active components were analyzed to construct a small molecule network map to explore the multitarget properties of the main active components (Figure 3(b)). A total of 124 quercetin targets, 23 beta-sitosterol targets, 23 stigmasterol targets, 46 kaempferol targets, 46 luteolin targets, 32 tanshinone IIA targets, and 27 naringenin targets were found.

### 3.5. Construction and Analysis of Protein-Protein Interaction Network

Based on the topological analysis, the target data generated from the STRING website was input into the Cytoscape 3.8.0 software. Greater than or equal to the median value was used as a filtering criterion, and the final topological parameter analysis yielded 18 nodes and 192 edges on the way to the PPI network, and STAT3, MAPK1, RELA, IL6, TNF, ESR1, and IL10 were identified as seven core targets (Table 2 and Figure 4).

### 3.6. GO Enrichment Analysis

The common drug-disease targets were input into the *R* language bioconductor package, and the GO and KEGG analyses were performed. The GO enrichment analysis included molecular function, biological pathway function, and cellular component. A bar chart was created using the top 10 entries (Figure 5), with the lower the bar, the smaller the P. Among them, the target protein molecular functions primarily focused on nuclear receptor activity, ligand activation, cytokine activity, DNA-binding transcription factor binding, and RNA polymerase II-specific DNA-binding transcription factor binding; cell composition, including membrane rafts, membrane microdomains, membrane regions, plasma membrane rafts, and postsynaptic membrane components; and biological processes, including responses to reactive oxygen species, drugs, lipopolysaccharides, and oxidative stress.

### 3.7. KEGG Analysis

Based on the gene ratios, the top 20 highly enriched pathways were screened (Table 3, Figures 6(a) and 6(b)). These 20 pathways, *P*-values from the KEGG enrichment analysis, and the associated targets and compounds were selected to develop a compound-target-pathway network using the Cytoscape 3.8.0 software (Figure 6(c)), containing 161 nodes and 671 edges. Obesity and diabetes treatment using the Huanglian Huazhuo capsules was via multiple pathways associated with various pathways, such as AGE-RAGE signaling pathway, fluid shear stress and atherosclerosis, HIF-1 signaling pathway, IL-17 signaling pathway, and TNF signaling pathway in diabetes complications. We also visualized the distribution of key targets in the most relevant path (Figure 7).

### 3.8. Prediction of the Binding Ability of the Huanglian Huazhuo Capsule Core Components to the Target Using Molecular Docking Technique

Molecular docking is a theoretical simulation method to examine the interaction between molecules and predict their binding mode and affinity. The top three target proteins and small molecules were screened for docking. Generally, the lower the energy required for ligand-molecule binding, the easier the docking success. If the binding energy is < 0 kcal/mol^−1^, the molecules bind by themselves (Table 4, Figure 8). The molecular docking results are shown in Figure 9. Hydrophobic small molecules and target protein active cavity form stable complexes via hydrogen bonding. In this study, tanshinone IIA showed strong binding activity with STAT3, MAPK1, IL6, and IL10, suggesting these as candidate drug molecules. Molecular docking techniques provide a strategy to assess the binding mode between herbal compounds and disease-related targets. However, potential herbal compounds require experimental validation.

## 4. Discussion

DM is a common chronic disease with increasing annual incidence. The number of patients with T2DM primarily characterized by insulin resistance is increasing [1]. Therefore, active intervention is required for the prognosis of T2DM. Currently, no specific drugs exist for T2DM treatment, bringing the clinical focus to glycemic control. Furthermore, the ideal efficacy of pure Western medical treatment is difficult to obtain, and new treatment methods are needed. Nevertheless, the positive role of Chinese medicine in diabetes prevention and treatment has been affirmed [6].

The Huanglian Huazhuo capsule removes phlegm, accumulation, dampness, and blood stasis and invigorates spleen. Among them, Huanglian and Huangbai removes heat and dampness and releases fire and detoxify; Shanzha digests and removes accumulation, strengthens stomach, and removes stasis by eliminating Qi; Zhiqiao detoxifies and removes turbidity; and Danshen promotes blood circulation and removes blood stasis. However, the bioactive compounds of the Huanglian Huazhuo capsules and their mechanisms of action against obese T2DM remain unclear. Therefore, the potential targets and mechanisms of action of the Huanglian Huazhuo capsules were identified in obese T2DM cases using a network pharmacology strategy and molecular docking.

A total of 88 active compounds from the TCMSP database were screened for the Huanglian Huazhuo capsules. Furthermore, 1056 obese T2DM disease targets were obtained from the geographic database. Hence, 108 putative Huanglian Huazhuo capsule-obese T2DM targets were identified. Based on the degree in the drug-component-target-disease network, the top seven active compounds of the Huanglian Huazhuo capsule were quercetin, beta-sitosterol, stigmasterol, kaempferol, luteolin, tanshinone IIA, and naringenin. Their effectiveness is supported by previous studies. Reportedly, quercetin attenuates lipid peroxidation, platelet aggregation, and capillary permeability and contains anti-inflammatory effects with therapeutic efficacy in obesity and T2DM [23]. Beta-sitosterol ameliorates the IKK*β*/NF-*κ*B and c-Jun-N-terminal kinase signaling pathways in the adipose tissue by downregulating inflammatory events, thereby inhibiting obesity-induced insulin resistance [24]. Stigmasterol and phytosterol-rich diets control glucolipid metabolism and insulin resistance [25]. Kaempferol increases lipid metabolism by downregulating PPAR-*γ* and SREBP-1c, thereby reducing adipose tissue accumulation and improving hyperlipidemia in mice with obesity and diabetes [26]. Luteolin attenuates neuroinflammation, oxidative stress, and neuronal insulin resistance in the mouse brain and normalizes blood adipocytokine levels [27]. Tanshinone IIA improves hepatic steatosis by inhibiting excess endoplasmic reticulum stress, endoplasmic reticulum stress-induced apoptosis, and hepatic steatosis [28]. Naringenin promotes adipose tissue in insulin receptor expression, GLUT4, lipocalin, and antidiabetic effects [29]. The strength of the protein gene role in the entire network is proportional to the degree value, and the protein genes with larger degree values play a significant role [30]. STAT3, MAPK1, RELA, IL6, TNF, ESR1, and IL10 were the seven core targets identified by the degree in the PPI network.

The KEGG and GO functional analyses showed that the effect of the Huanglian Huazhuo capsule in obese T2DM is associated with many biological processes, including inflammatory, lipopolysaccharide, and oxidative stress responses. In this study, the targets were enriched for lipid and inflammatory response pathways, such as HIF-1, IL-17, and TNF signaling pathways. HIF-1 reportedly promotes changes in the adipose tissues of patients with obesity, leading to the inhibition of adipocyte differentiation, adipocyte dysfunction, inflammation, insulin resistance, and T2D [31]. An adipose tissue from patients with obesity and T2D produced specific enrichment of CD4+ T cells for IL-17 and IL-22, which is pathologically relevant to obesity-induced T2D [32]. Furthermore, TNF is associated with obesity and T2D and correlates with glycated hemoglobin [33].

Subsequently, seven key target proteins, such as STAT3, MAPK1, RELA, IL6, TNF, ESR1, IL10, and active compounds, including quercetin, beta-sitosterol, stigmasterol, kaempferol, luteolin tanshinone IIA, naringenin, were evaluated using molecular docking techniques. The binding affinities ranged from −5.1 to −9.0 kcal/mol, indicating that all targets possibly had good docking ability with the active compounds. The result suggests that these compounds may contribute to the effectiveness of the Huanglian Huazhuo capsules in obese T2DM treatment. Chronic low-grade inflammation with elevated levels of nonspecific inflammatory factors, T2DM is an important factor in T2DM development and its complications [34]. The major signaling pathways involved in the inflammatory response include the NF-ΚB, JAK/STAT, MAPK, and PI3K/AKT signaling pathways. Obesity caused by T2MD was treated using the Huanglian Huazhuo capsule mainly through the MAPK, PI3K/AKT, and Wnt signaling pathways (Figure 7). MAPK1, IL6, IL10, STAT3, and ESR1, which bind to small molecules, were stable (Figure 8). MAPK1 is one of the crucial molecules in the MAPK signaling pathway, and its activation regulates the downstream inflammatory response and glucose and lipid metabolisms, as cytokines involved in inflammation and immunosuppression [35, 36]. IL6 and IL10 are regulated by the PI3K/AKT, tgf-*β*, and Wnt signaling pathways, and they closely associate with the inflammatory signaling pathway [37–39]. These results are consistent with our finding that the Huanglian Huazhuo capsules treat obese T2DM via the inflammatory response pathway. However, in vitro experiments are required to validate these results.

However, the present study has some limitations. First, bioactive compounds and target data were retrieved from the literature and databases; hence, the reliability and accuracy of the predictions depend on the data quality. The active compounds in the Huanglian Huazhuo capsules can be analyzed using the lC/MS technique. In addition, metabolomics and pharmacokinetic studies may be advantageous. Second, data mining methods that require clinical trials and animal studies to confirm these findings were used.

## 5. Conclusions

It is the first time that the pharmacological and molecular mechanisms of action of the Huanglian Huazhuo capsule have been systematically explored to treat obese T2DM using network pharmacology and molecular docking techniques. These bioinformatics and computational analyses suggest that quercetin, beta-sitosterol, stigmasterol, and kaempferol are possibly the main active compounds of the Huanglian Huazhuo capsule in obese T2DM treatment. In addition, the Huanglian Huazhuo capsule could treat obese T2DM by reducing pathological damage, inflammatory response, and oxidative stress via various pathways, such as HIF1, IL-17, and TNF. Overall, the present study focused on the multicomponent and multipathway nature and mechanism of action of the Huanglian Huazhuo capsule. These findings can guide the application and further develop the Huanglian Huazhuo capsules in obese T2DM treatment.

## Figures and Tables

**Figure 1:** Screening of common targets for the Huanglian Huazhuo capsule-obese T2DM. (a) The differential gene volcano plot shows gene distribution in the disease samples. Red and green represent upregulated and downregulated genes, respectively, and black indicates no significant difference. (b) The heat map shows the expression patterns of 28 DEGs. Columns correspond to samples, and rows correspond to genes.

**Figure 2:** Venn diagram of the Huanglian Huazhuo capsule corresponding to target and disease corresponding to target intersection. Green represents the number of targets of the active components of the drug, and pink represents the number of disease-related genes, which are 108 cross-targeted genes.

**Figure 3:** (a) In the “drug-component-target-disease” network, the pink circles represent the Huanglian Huazhuo capsules, the blue rectangles represent drugs, the green diamonds represent drug compounds, the purple circles represent diseases, and the blue triangles represent target proteins. (b) In the small molecule network plot, blue represents quercetin and its corresponding target, purple represents beta-sitosterol and its corresponding target, cyan represents stigmasterol and its corresponding target, red represents kaempferol and its corresponding target, pink represents luteolin and its corresponding target, red represents tanshinone IIA and its corresponding targets, and green represents naringenin and its corresponding targets.

**Figure 4:** Topological screening process of the PPI network. A total of 85 common targets were screened using degree centrality (DC), betweenness centrality (BC), and closeness centrality (CC), and seven core targets were obtained.

**Figure 5:** GO enrichment analysis. (a) Histogram of biological process category terms in the GO enrichment analysis. (b) Bubble diagram of biological process category terms in the GO enrichment analysis.

**Figure 6:** KEGG enrichment analysis and critical path network construction. (a) Histogram of the top 20 pathways based on KEGG enrichment analysis. (b) Bubble diagram of the top 20 pathways based on KEGG enrichment analysis. (c) Compound-target-pathway network associated with the mechanism of the Huanglian Huazhuo capsule for obese T2DM treatment. Purple nodes represent targets, dark green nodes represent compounds, and light green nodes represent pathways.

**Figure 7:** Distribution of key targets in the most relevant paths.

**Figure 8:** Thermogram of molecular docking fractions. Binding energy of key targets and herbal active compounds (kcal/mol).

**Figure 9:** Docking patterns of key targets and specific active compounds. Tanshinone IIA-STAT3 (a), tanshinone IIA-MAPK1 (b), luteolin-RELA (c), tanshinone IIA-IL6 (d), stigmasterol-TNF (e), quercetin-ESR1 (f), and tanshinone IIA-IL10 (g).

**Table 1:** Active ingredients in the Huanglian Huazhuo capsules.

Name	Pubchem ID	Compound	OB	DL%
Danshen	124416	MOL0016011,2,5,6-t	38.75	0.36
Danshen	5281330	MOL001659Poriferas	43.83	0.76
Danshen	457801	MOL001771Poriferas	36.91	0.75
Danshen	68081	MOL001942Isoimpera	45.46	0.23
Danshen	94162	MOL002222Sugiol	36.11	0.28
Danshen	128994	MOL002651Dehydrota	43.76	0.4
Danshen	64982	MOL002776Baicalin	40.12	0.75
Danshen	54711004	MOL000569Digallate	61.85	0.26
Danshen	5280445	MOL000006luteolin	36.16	0.25
Danshen	11593487	MOL0070365,6-dihyd	33.77	0.29
Danshen	135872	MOL0070412-isoprop	40.86	0.23
Danshen	1.01E+08	MOL0070453*α*-hydro	44.93	0.44
Danshen	14609851	MOL0070494-methyle	34.35	0.23
Danshen	95223221	MOL0070502-(4-hydr	62.78	0.4
Danshen	14609847	MOL007058formyltan	73.44	0.42
Danshen	10995850	MOL0070593-beta-Hy	32.16	0.41
Danshen	105118	MOL007061Methylene	37.07	0.36
Danshen	16090911	MOL007063Przewalsk	37.11	0.65
Danshen	16102114	MOL007064Przewalsk	110.32	0.44
Danshen	622085	MOL007068Przewaqui	62.24	0.41
Danshen	56967683	MOL007069Przewaqui	55.74	0.4
Danshen	10470747	MOL007070(6S,7R)-6	41.31	0.45
Danshen	126073	MOL007071Przewaqui	40.31	0.46
Danshen	163263	MOL007077Sclareol	43.67	0.21
Danshen	124268	MOL007079Tanshinal	52.47	0.45
Danshen	3083515	MOL007081Danshenol	57.95	0.56
Danshen	3083514	MOL007082Danshenol	56.97	0.52
Danshen	389885	MOL007085Salvileno	30.38	0.38
Danshen	160254	MOL007088Cryptotan	52.34	0.4
Danshen	127172	MOL007093Dan-shenx	38.88	0.55
Danshen	1.02E+08	MOL007094Danshensp	50.43	0.31
Danshen	15690458	MOL007098Deoxyneoc	49.4	0.29
Danshen	34754315	MOL007100Dihydrota	38.68	0.32
Danshen	11425923	MOL007101Dihydrota	45.04	0.36
Danshen	1.02E+08	MOL007105Epidanshe	68.27	0.31
Danshen	442027	MOL007107C09092	36.07	0.25
Danshen	626608	MOL007108Isocrypto	54.98	0.39
Danshen	44425166	MOL007111Isotanshi	49.92	0.4
Danshen	3034394	MOL007115Manool	45.04	0.2
Danshen	5319835	MOL007119Miltionon	49.68	0.32
Danshen	5319836	MOL007120Miltionon	71.03	0.44
Danshen	10086184	MOL007121Miltipolo	36.56	0.37
Danshen	160142	MOL007122Miltirone	38.76	0.25
Danshen	15690458	MOL007124Neocrypto	39.46	0.23
Danshen	389888	MOL007125Neocrypto	52.49	0.32
Danshen	10062187	MOL0071271-methyl-	34.72	0.37
Danshen	30428202	MOL007130prolithos	64.37	0.31
Danshen	65035	MOL007132(2R)-3-(3	109.38	0.35
Danshen	11530200	MOL007141Salvianol	45.56	0.61
Danshen	24177556	MOL007142Salvianol	43.38	0.72
Danshen	389885	MOL007143Salvileno	32.43	0.23
Danshen	389885	MOL007145Salviolon	31.72	0.24
Danshen	5321620	MOL007151Tanshindi	42.67	0.45
Danshen	126072	MOL007152Przewaqui	42.85	0.45
Danshen	164676	MOL007154Tanshinon	49.89	0.4
Danshen	9926694	MOL007155(6S)-6-(h	65.26	0.45
Danshen	149138	MOL007156Tanshinon	45.64	0.3
Huangbai	2353	MOL001454Berberine	36.86	0.78
Huangbai	72322	MOL001458Coptisine	30.67	0.86
Huangbai	5320517	MOL002641Phellavin	35.86	0.44
Huangbai	98608	MOL002644Phellopte	40.19	0.28
Huangbai	128994	MOL002651Dehydrota	43.76	0.4
Huangbai	65752	MOL002662Rutaecarp	40.3	0.6
Huangbai	6760	MOL002663Skimmiani	40.14	0.2
Huangbai	2703	MOL002666Cheleryth	34.18	0.78
Huangbai	5280794	MOL000449Stigmaste	43.83	0.76
Huangbai	20055073	MOL002668Worenine	45.83	0.87
Huangbai	193148	MOL002670Cavidine	35.64	0.81
Huangbai	222284	MOL000358Beta-sito	36.91	0.75
Huangbai	5319198	MOL000622Magnogran	63.71	0.19
Huangbai	19009	MOL000785Palmatine	64.6	0.65
Huangbai	4970	MOL000787Fumarine	59.26	0.83
Huangbai	440229	MOL000790Isocorypa	35.77	0.59
Huangbai	5280343	MOL000098Quercetin	46.43	0.28
Huangbai	193876	MOL001131Phellamur	56.6	0.39
Huangbai	21171	MOL001455(S)-canad	53.83	0.77
Huangbai	457801	MOL001771Poriferas	36.91	0.75
Huangbai	72703	MOL002894Berberrub	35.74	0.73
Huangbai	3084288	MOL006422Thalifend	44.41	0.73
Huanglian	5319198	MOL000622Magnogran	63.71	0.19
Huanglian	5280343	MOL000098Quercetin	46.43	0.28
Huanglian	19009	MOL000785Palmatine	64.6	0.65
Huanglian	72703	MOL002894Berberrub	35.74	0.73
Huanglian	443422	MOL002903(R)-canad	55.37	0.77
Huanglian	160876	MOL002897Epiberber	43.09	0.78
Huanglian	2353	MOL001454Berberine	36.86	0.78
Huanglian	11066	MOL002904Berlambin	36.68	0.82
Huanglian	72322	MOL001458Coptisine	30.67	0.86
Huanglian	20055073	MOL002668Worenine	45.83	0.87
Shanzha	5281654	MOL000354Isorhamne	49.6	0.31
Shanzha	222284	MOL000359Sitostero	36.91	0.75
Shanzha	5280863	MOL000422Kaempfero	41.88	0.24
Shanzha	5280794	MOL000449Stigmaste	43.83	0.76
Shanzha	182232	MOL000073Ent-epica	48.96	0.24
Shanzha	5280343	MOL000098Quercetin	46.43	0.28
Zhiqiao	6450230	MOL013381Marmin	38.23	0.31
Zhiqiao	72281	MOL002341Hespereti	70.31	0.27
Zhiqiao	222284	MOL000358Beta-sito	36.91	0.75
Zhiqiao	932	MOL004328Naringeni	59.29	0.21
Zhiqiao	72344	MOL005828Nobiletin	61.67	0.52

**Table 2:** Seven core targets.

PDB ID	Gene name	Gene symb	Protein name	Degree
5AX3	STAT3	P40763	Signal transducer and activator of transcription 3	18
7.00E+75	MAPK1	P28482	Transcription factor p65	16
7LEU	RELA	Q04206	Transcrip	14
1IL6	IL6	P05231	Interleuk	12
7QLF	TNF	P01375	Tumor nec	11
7RS8	ESR1	P03372	Estrogen	9
1ILK	IL10	P22301	Interleuk	9

**Table 3:** KEGG enrichment analysis of key genes.

ID	Description	GeneID	Count
hsa04933	AGE-RAGE signaling pathway in diabetic complications	MMP2, TNF, BCL2, RELA, AKT1, VEGFA, MAPK1, IL6, STAT1, F3, ICAM1, IL1B, CCL2, SELE, VCAM1, CXCL8, PRKCB, NOS3, THBD, SERPINE1, COL1A1, COL3A1, STAT3, EDN1, MAPK8	25

hsa05418	Fluid shear stress and atherosclerosis	MMP2, MMP9, TNF, BCL2, KDR, RELA, AKT1, VEGFA, TP53, HMOX1, CAV1, ICAM1, IL1B, CCL2, SELE, VCAM1, NOS3, PLAT, THBD, IFNG, GSTP1, NFE2L2, NQO1, GSTM1, EDN1, IKBKB, MAPK8	27

hsa05417	Lipid and atherosclerosis	RXRA, PPARG, MMP9, TNF, BCL2, CASP9, MMP3, RELA, AKT1, MAPK1, IL6, TP53, MMP1, CYP1A1, ICAM1, IL1B, CCL2, SELE, VCAM1, CXCL8, NOS3, NFE2L2, CD40LG, GSK3B, STAT3, OLR1, IKBKB, MAPK8, APOB	29

hsa04066	HIF-1 Signaling pathway	NOS2, BCL2, RELA, EGFR, AKT1, VEGFA, MAPK1, EGF, IL6, HIF1A, ERBB2, HMOX1, PRKCB, NOS3, SERPINE1, IFNG, INSR, HK2, STAT3, EDN1, TIMP1	21

hsa04657	IL-17 Signaling pathway	PTGS2, MMP9, TNF, IL4, MMP3, RELA, MAPK1, IL6, MMP1, IL1B, CCL2, CXCL8, IFNG, CXCL10, GSK3B, IKBKB, MAPK8	17

hsa04668	TNF Signaling pathway	PTGS2, MMP9, TNF, MMP3, RELA, AKT1, MAPK1, IL6, ICAM1, IL1B, CCL2, SELE, VCAM1, CXCL10, EDN1, IKBKB, MAPK8, CREB1	18

hsa05215	Prostate cancer	AR, MMP9, BCL2, CASP9, MMP3, RELA, EGFR, AKT1, MAPK1, EGF, TP53, ERBB2, PLAT, GSTP1, GSK3B, IKBKB, CREB1	17

hsa05207	Chemical carcinogenesis-receptor activation	ESR1, AR, RXRA, ADRB2, CYP3A4, CYP1A2, PGR, ADRB1, BCL2, RELA, EGFR, AKT1, VEGFA, MAPK1, EGF, CYP1A1, PRKCB, BIRC5, PPARA, GSTM1, STAT3, CREB1	22

hsa05142	Chagas disease	NOS2, TNF, RELA, AKT1, MAPK1, IL10, IL6, IL1B, CCL2, CXCL8, IL2, SERPINE1, IFNG, IKBKB, MAPK8	15

hsa04931	Insulin resistance	TNF, RELA, AKT1, IL6, PRKCB, NOS3, SLC2A4, INSR, PPARA, GSK3B, STAT3, IKBKB, MAPK8, SREBF1, CREB1	15

hsa05212	Pancreatic cancer	CASP9, RELA, EGFR, AKT1, VEGFA, MAPK1, EGF, TP53, STAT1, ERBB2, STAT3, IKBKB, MAPK8	13

hsa05161	Hepatitis B	MMP9, TNF, BCL2, CASP9, RELA, AKT1, MAPK1, IL6, TP53, STAT1, CXCL8, PRKCB, BIRC5, STAT3, IKBKB, MAPK8, CREB1	17

hsa05144	Malaria	TNF, IL10, IL6, ICAM1, IL1B, CCL2, SELE, VCAM1, CXCL8, IFNG, CD40LG	11

hsa04151	PI3K-Akt signaling pathway	RXRA, IL4, BCL2, CASP9, KDR, RELA, EGFR, AKT1, VEGFA, MAPK1, EGF, IL6, TP53, ERBB2, NOS3, IL2, COL1A1, INSR, SPP1, IGF2, GSK3B, IKBKB, CREB1	23

hsa05219	Bladder cancer	MMP2, MMP9, EGFR, VEGFA, MAPK1, EGF, TP53, MMP1, ERBB2, CXCL8	10

hsa04926	Relaxin signaling pathway	NOS2, MMP2, MMP9, RELA, EGFR, AKT1, VEGFA, MAPK1, MMP1, NOS3, COL1A1, COL3A1, EDN1, MAPK8, CREB1	15

hsa05160	Hepatitis C	RXRA, TNF, CASP9, RELA, EGFR, AKT1, MAPK1, EGF, TP53, STAT1, IFNG, PPARA, CXCL10, GSK3B, STAT3, IKBKB	16

hsa05145	Toxoplasmosis	NOS2, TNF, BCL2, CASP9, RELA, AKT1, MAPK1, IL10, STAT1, IFNG, CD40LG, STAT3, IKBKB, MAPK8	14

hsa01521	EGFR tyrosine kinase inhibitor resistance	BCL2, KDR, EGFR, AKT1, VEGFA, MAPK1, EGF, IL6, ERBB2, PRKCB, GSK3B, STAT3	12

hsa05167	Kaposi sarcoma-associated herpesvirus infection	PTGS2, CASP9, RELA, AKT1, VEGFA, MAPK1, IL6, TP53, HIF1A, STAT1, ICAM1, CXCL8, GSK3B, STAT3, IKBKB, MAPK8, CREB1	17

**Table 4:** Binding energy of active ingredients to target proteins.

Compound	Chemical formula	Relative molecular weight g/mol	Binding energy / kcal mol^–1^					
			STAT3	MAPK1	RELA	IL6	TNF	ESR1	IL10
Quercetin	C15H10O7	302.23	−7.4	−8.9	−6.8	−6.9	−5.2	−8.1	−6.7
Beta-sitosterol	C29H50O	414.7	−7.0	−8.2	−6.3	−6.6	−5.3	−7.3	−7.8
Stigmasterol	C29H48O	412.7	−7.0	−8.6	−6.4	−6.3	−6.4	−7.8	−8.5
Kaempferol	C15H10O6	286.24	−7.4	−8.5	−6.7	−6.8	−5.0	−7.9	−7.0
Luteolin	C15H10O6	286.24	−7.7	−8.8	−6.9	−7.2	−5.3	−8.0	−6.9
Tanshinone IIA	C19H18O3	294.3	−8.2	−9.0	−6.5	−7.8	−6.0	−8.0	−8.6
Naringenin	iC15H12O5	272.25	−7.3	−8.3	−6.7	−7.0	−5.1	−7.7	−6.9

## Data Availability

The data in the study are obtained from TCMSP, CNKI, PubMed, GEO, RSCB PDB, and PubChem.
